The article "Design of Public Building Space in Smart City Based on Big Data" was published in 2022. Journal: J Environ Public Health.

# Design of Public Building Space in Smart City Based on Big Data

**DOI:** 10.1155/2022/4733901

**Published:** 2022-08-25

**Authors:** Wei Wang

**Affiliations:** Xinyang College of Fine Arts and Design, Xinyang, Henan 464000, China

## Abstract

In order to improve the geometric form space composition and color planning analysis ability of smart city public buildings, a big data based smart city public building space design method is proposed. The method of combining computer vision detection and remote sensing detection is adopted to realize the detection of big data characteristics of spatial combination at the aesthetic level of building structure, and the difference distribution model of spatial composition parameters of building geometry is constructed. Extract the feature quantity of urban architectural integration form elements, and build the big data GIS information base of spatial combination at the aesthetic level of architectural structure according to the analysis results of intelligent parameters, so as to realize the spatial design of the intelligent urban public buildings. The test shows that the application of this method improves the geometric form space composition and color planning ability of smart city public buildings and can realize high-precision spatial combination big data extraction of architectural structure aesthetics in a large area. At the same time, this method can ensure the relative independence of space and meet the requirements of use and management.

## 1. Introduction

In the process of China's urban development, the high population density and low per capita land resources inevitably lead to the high-density development of urban central areas, and all kinds of social resources and development opportunities are also concentrated in urban central areas, which in turn further attracts people around the city to gather, thus bringing congestion and environmental deterioration in urban central areas. The public space is constantly eroded, and the central area is gradually becoming indifferent and mechanical. The scale of high-rise buildings is obviously separated from that of people, and the bottom of high-rise buildings becomes a negative space in the city [1]. The indifferent building facade and the lack of public space limit the emergence of urban activities, and people huddle inside the buildings, leaving the city with only their hurried backs. The building has also developed from the horizontal to the centralized and high-altitude direction in the past. The high-altitude part is difficult to touch the ground and isolated from the urban space, thus becoming an isolated island in the city. At the same time, with the increase of volume, it is inevitable that more demands will be extended, resulting in mixed functions. However, the design of architectural space lags behind the demand, which leads to the cramped space, difficult to use, and even potential safety hazards [2, 3].

The article "Design of Public Building Space in Smart City Based on Big Data" was published in 2022. Journal: J Environ Public Health.

In order to solve these problems, many city managers choose to build new urban areas. However, because the concept of urban planning and architectural design has not changed, the construction of new urban areas will easily lead to the scarcity of population in the early stage and the overcrowding in the later stage, making it difficult to jump out of the old road of urban development [4, 5]. Therefore, it is necessary to study the spatial composition and color planning design method of public buildings in smart cities, analyze the remote sensing parameters under the spatial distribution of public buildings in smart cities by combining the remote sensing impact identification, and carry out the spatial composition and color planning design of public buildings in smart cities by combining the image feature analysis method, so as to establish the remote sensing information database of spatial composition and color planning design of public buildings in smart cities [6–8]. Using the method of GIS information base construction and remote sensing parameter identification, it is of great significance to detect and track the change of geometric spatial information of public buildings in smart cities in real time, and to study the geometric spatial composition and color planning and design methods of public buildings in smart cities, which will promote urban construction and urban building development [9, 10].

At present, in the planning and design of smart city public buildings, the main methods are the identification method of smart city public buildings' geometric space configuration parameters based on synthetic aperture radar [11, 12], the identification method of smart city public buildings' geometric space configuration and color planning and design based on echo signal detection, and the image parameter identification method based on SAR. Combined with the distribution characteristics and contour parameter distribution of smart city public buildings, spatial image filtering and remote sensing detection are adopted to carry out the geometric space configuration and color planning and design of smart city public buildings. In reference [13], a method of extracting smart city public buildings from SAR images by combining speckle suppression with multi-resolution topological analysis is proposed. In the anisotropic diffusion distribution domain of speckle suppression, a gradient analysis model of spatial combination big data at the architectural structure aesthetic level is established, and the high-score SAR images are verified and analyzed by combining spectral analysis and image denoising. However, this method has poor ability to identify and judge discontinuities. In reference [14], multispectral optical remote sensing images are used to design the extraction model of the geometric form space composition of public buildings in smart cities. According to the similar reflection characteristics between ground objects and the geometric form space composition of public buildings in smart cities, the geometric form space composition characteristics of public buildings in smart cities are analyzed and identified. However, this method has poor performance in the spatial structure layout design of large-scale urban buildings [15, 16].

The article "Design of Public Building Space in Smart City Based on Big Data" was published in 2022. Journal: J Environ Public Health.

In view of the above problems, this paper proposes a smart city public building space design method based on big data. Firstly, the method of combining computer vision detection and remote sensing detection is used to detect the geometric form and spatial structure of public buildings in smart cities. Then, the big data analysis model of spatial combination at the aesthetic level of building structure is established, and the big data parameter identification of spatial combination at the aesthetic level of building structure is realized by combining GIS remote sensing information feature analysis and image feature detection. Finally, the experimental test shows the effectiveness and superiority of this method.

## 2. Theoretical Analysis of Big Data Technology

Full-scale extraction of big data is similar to data migration or data replication. It extracts the data from the data source intact from the database and converts it into a format that the ETL tools can recognize. Total extraction is relatively simple. Incremental extraction only extracts new or modified data from the table to be extracted in the database since the last extraction. In the use of ETL, incremental extraction is more widely used than full extraction. In the process of big data application, it is necessary to control the accuracy of data extraction, convert the required data in the system, and capture it accurately according to a certain frequency. The spatial combination of big data in architectural aesthetics can be completely loaded by deleting and inserting the whole table. Before extracting data every time, you can delete the target table data first, and load the data completely new when extracting. This method actually equates incremental extraction with full extraction. For spatial combination data with a small amount of data, the time cost of total extraction is less than the algorithm and conditional cost of incremental extraction. Hierarchical storage of data is carried out according to data warehouse. On the one hand, this architecture is related to the way of data pulling, and on the other hand, it is for hierarchical abstract processing of data. The data warehouse is divided into three layers, namely, posting source layer, historical storage layer, and data model layer. Sticking to the source layer means that the data is consistent with the data of the source system, which can ensure that the data source of the data warehouse is real, and at the same time, it is convenient to check after the data goes wrong. For the data of the source system extracted by the attached source layer, the method of total extraction can be adopted. The history layer refers to the historical data, which is equivalent to a copy of the business library as of a certain time. The history layer can completely copy all the data in the business database and effectively store the resources. The data layer refers to the level of dimension modeling according to the business system, which is based on a certain business application to improve the data application effect. Big data technology has the characteristics of accurate and available data, traceable history, safety, and controllability.  Figure 1 shows the big data processing flow.

The article "Design of Public Building Space in Smart City Based on Big Data" was published in 2022. Journal: J Environ Public Health.

## 3. Model Mechanism and Index Analysis of Public Building Space Design

### 3.1. Model Mechanism

In the planning and design of the geometric form and color of public buildings in smart cities based on the spatial combination big data of architectural structure aesthetics, the multi-band water index (MBWI) feature analysis method is adopted to construct the MBWI monitoring and analysis model, and the GIS remote sensing monitoring is adopted. The detected images are distributed in several Landsat 8, Sentinel 2 and GF-1 images. The high-resolution remote sensing monitoring method is adopted to analyze the spatial information characteristics of the geometric form of public buildings in smart cities, and a global multi-scale feature detection model of the spatial information of the geometric form of public buildings in smart cities is established. Combined with the dynamic feature distribution of remote sensing GIS of the original images, a long-distance global information capture method is adopted [17–19]. The GIS information base is established. Through the feature extraction of high-resolution GIS remote sensing images, the images are segmented in the shallow features and fine-grained deep features of the geometric space of public buildings in smart cities [20, 21]. Based om = *n* feature extraction and fusion, the multi-dimensional scale analysis models with different spectral lengths are established. The weighted sum of features of all positions is used to evaluate the spatial information of public buildings in smart cities by map information theory in different functional blocks. In the basic geographic information database, the full-automatic information loading method is adopted to establish the spatial information distribution rules of public buildings in smart cities under different environments, including the spatial composition of public buildings in smart cities and the spatial composition of public buildings in marine smart cities. Therefore, using the normalized analysis method of spatial composition index of public buildings in smart cities, the difference distribution model of spatial composition parameters of public buildings in smart cities with the change of spatial combination of architectural structure aesthetics is constructed, and the spatial planning and color aesthetic positioning of public buildings in smart cities are carried out by the method of joint characteristic analysis of urban development and spatial layout. The technical realization model is shown in Figure 2.

The article "Design of Public Building Space in Smart City Based on Big Data" was published in 2022. Journal: J Environ Public Health.

Based on Figure 2, the spatial index characteristics of intelligent urban public buildings can be divided into the following parts: shadow, greening, energy saving, ground transportation, underground pipe network, and urban blocks. Feature detection is realized through the blue band, green band, red band, near-infrared band, and short wave of GIS technology.

According to the technical road map in Figure 2, this paper analyzes the spatial information changes of public buildings in smart cities under different spatial composition indexes of public buildings in short-wave near-infrared band and dual-band, and establishes a GIS remote sensing information monitoring database of spatial information changes of public buildings in smart cities. Through the analysis of spatial composition parameters of public buildings in smart cities, the spatial composition indexes of public buildings in smart cities are carried out under different ground objects [22].

### 3.2. Analysis of Spatial Composition Index of Urban Public Buildings' Geometric Form

#### 3.2.1. Theoretical Basis of Computer Vision

Computer vision is to use various imaging systems to replace visual organs as input sensitive means, and computers to replace the brain to complete processing and interpretation. The ultimate research goal of computer vision is to enable computers to observe and understand the world through vision like people, and have the ability to adapt to the environment independently.

The article "Design of Public Building Space in Smart City Based on Big Data" was published in 2022. Journal: J Environ Public Health.

Computer vision analyzes the images and then creates a numerical representation of what they “see” using convolutional neural networks (CNNs). CNN is a kind of artificial neural network, which uses convolution layer to filter useful information from input. Convolution operation needs to use input data (feature map) and convolution kernel (filter) to generate converted feature map. The convolution layer filter can be modified according to the learning parameters to extract the most useful information for a specific task. The convolution network can be automatically adjusted according to the task to find the most important features. When performing a general object recognition task, CNN will filter the shape information of the object. However, in the task of identifying birds, CNN will extract the color information of birds. This is because the CNN believes that different types of objects have different shapes, and for different types of birds, their colors may be more different than their shapes.

Segmentation: image segmentation refers to classifying pixels into specific categories, such as cars, roads, or pedestrians. It is widely used in autonomous vehicle applications (including NVIDIA drive ™ Software stack) for displaying roads, cars, and people. You can think of it as a visualization technology that makes it easier for people to understand the work of computers.

Classification: image classification is used to determine the content in the image. For example, after training, neural networks can recognize dogs or cats, or many other things, and have high accuracy.

Detection: through image detection, the computer can locate the position of the object. In many applications, CNN will set a rectangular bounding box around the relevant area to completely include the objects. The detector may also be trained to detect the position of the vehicle or person in the image.

Computer vision is to use various imaging systems to replace visual organs as input sensitive means, and computers to replace the brain to complete processing and interpretation. The ultimate research goal of computer vision is to enable computers to observe and understand the world through vision like human beings, and have the ability to adapt to the environment independently.

To sum up, the main principle of computer vision is to realize the global motion compensation of the background through feature point matching on the basis of collecting the geometric shape spatial sequence images of smart city public buildings.

#### 3.2.2. Analysis of Spatial Composition Index of Building Geometry

By constructing the spatial index analysis model of public buildings in smart cities, and combining with the spatial parameter distribution of public buildings in smart cities, the spatial index characteristics of public buildings in smart cities are analyzed. The data sources are Landsat 8, Sentinel 2, and GF-1, and the sampling objects of surface reflectivity are: spatial structure of public buildings in smart cities, spatial features of public buildings, etc. According to the ratio of different bands and green bands of each land object, set up a six-element inequality group, analyze the information changes of geometric form space composition index of public buildings in smart cities in different data sources, and analyze the similarity between reflection characteristics and geometric form space composition of public buildings in smart cities according to the differences between green bands and near-infrared bands, so as to construct your geometric form space composition index model of public buildings in smart cities, as shown in Figure 3.

The article "Design of Public Building Space in Smart City Based on Big Data" was published in 2022. Journal: J Environ Public Health.

On this basis, the feature quantity of the integrated form elements of urban buildings is extracted, and the formula model of spatial composition index of geometric form of public buildings in smart cities is constructed by connecting regional distribution, using the analysis method of spatial and geometric relationship among targets and combining with regression analysis.

(1) $$\begin{array}{c} Y=\left[\begin{array}{cccccc} x_{1} & x_{2} & x_{3} & x_{4} & x_{5} & x_{6} \end{array}\right]\left[\begin{array}{c} \rho_{1}\\ \rho_{2}\\ \rho_{3}\\ \rho_{4}\\ \rho_{5}\\ \rho_{6} \end{array}\right], \end{array}$$

where *Y* represents the spatial composition index distribution value of public buildings in smart cities, *x*_1_, *x*_2_,…, *x*_6_ represents the spectral coefficients of six bands obtained from the collected GIS remote sensing data, and *ρ*_1_, *ρ*_2_,…, *ρ*_6_ represents the reflectivity of different bands in the spatial composition index model parameters of public buildings in smart cities. By normalization, the spatial composition index distribution expression of public buildings in smart cities is divided by the green band, which can be transformed into:

(2) $$\begin{array}{c} \frac{Y}{\rho_{2}}=\left[\begin{array}{cccccc} x_{1} & x_{2} & x_{3} & x_{4} & x_{5} & x_{6} \end{array}\right]\left[\begin{array}{c} \frac{\rho_{1}}{\rho_{1}}\\ 1\\ \frac{\rho_{3}}{\rho_{2}}\\ \frac{\rho_{4}}{\rho_{2}}\\ \frac{\rho_{5}}{\rho_{2}}\\ \frac{\rho_{6}}{\rho_{2}} \end{array}\right]\\ =\left[\begin{array}{cccccc} x_{1} & x_{2} & x_{3} & x_{4} & x_{5} & x_{6} \end{array}\right]\left[\begin{array}{c} Q_{1}\\ Q_{2}\\ Q_{3}\\ Q_{4}\\ Q_{5}\\ Q_{6} \end{array}\right], \end{array}$$

where *Q*_1_, *Q*_2_,…, *Q*_6_ represent the ratio of blue band to green band, green band itself, red band to green band, near-infrared band to green band, short-wave near-infrared 1 to green band, and short-wave near-infrared 2 to green band, respectively [23, 24]. According to the geometric form spatial composition index of smart city public buildings obtained by formula (2), the spatial change characteristics of geometric form are identified by taking the band ratio as the research object and combining the GIS remote sensing monitoring results.

The article "Design of Public Building Space in Smart City Based on Big Data" was published in 2022. Journal: J Environ Public Health.

## 4. Recognition Algorithm of Spatial Variation Characteristics of Public Buildings in Smart Cities

### 4.1. Spatial Remote Sensing Image Processing of Public Building Geometry in Smart City

Combined with the local and global gray values of the geometric form space remote sensing images, the difference distribution model of the geometric form space composition parameters of the smart city public buildings with the change of the spatial combination of the architectural structure aesthetics is constructed [25, 26]. By solving the model, the gray difference values of different pixel feature points *c*_1_, *c*_2_ of GIS remote sensing images with spatial combination changes in architectural structure aesthetics are obtained, as shown in the following formula:

(3) $$\begin{array}{c} g\left(c_{1},c_{2}\right)=k\left(c_{1},c_{2}\right)⊗f\left(c_{1},c_{2}\right)+n, \end{array}$$

where ⊗ is convolution operator, *c*_1_, *c*_2_ are pixel feature point, *k*(*c*_1_, *c*_2_) is the difference information of original image, *f*(*c*_1_, *c*_2_) is the spatial distribution information of public building geometry in smart city captured in space or channel, and *n* is the prior noise of remote sensing GIS.

Based on the gray-scale difference value obtained by formula (3), the analysis process of spatial combination gray-scale value on the aesthetic level of building structure is designed, as shown in Figure 4.

By using the method of pyramid space pool module analysis, the spatial information variation of public buildings in smart cities is processed and detected in blocks. The multi-scale features of the input feature map are as follows:

(4) $$\begin{array}{c} C_{\text{mid}}=\sum_{i=-\infty }^{\infty }\sum_{j=0}^{N_{p}-1}p\left(t-iT_{s}\right)+q_{0}\exp\left(-\xi \rho \right). \end{array}$$

In the formula, *T*_*s*_ is the distribution coefficient of geometric features detected by remote sensing, *q*_0_ is edge similarity, *ξ* is weak correlation coefficient of spatial information of geometric features of public buildings in smart cities, *ρ* is image features in images, *t* is detection interval, *i* is edge noise reduction component, and *N*_*p*_ is detection error of public buildings in smart cities. Combined with the regional feature detection method, the fusion processing of GIS remote sensing images of spatial combination change in architectural structure aesthetics level is carried out. By using the method of connected region index, all connected regions are traversed, and the statistical feature quantity is expressed as follows:

(5) $$\begin{array}{c} x\left(t\right)=\sum_{m=1}^{M}\sum_{k=1}^{K\left(m\right)}w_{nk}s\left(t-T_{m}-\tau_{mk}\right)+v\left(t\right). \end{array}$$

In the above formula, *w*_*mk*_ is the characteristic component of extracting the information of the geometric form space of public buildings in smart cities, *T*_*m*_ is the reflectivity of near-infrared band, *τ*_*mk*_ is the geometric form space composition index of public buildings in smart cities, *v*(*t*) is the gray scale of images, and *K*(*m*) is the number of edge measurement points. Therefore, through the fuzzy infiltration of the space interface and the interactive changing parameters of the inner and outer spaces, the geometric space composition and color positioning of public buildings in smart cities can be detected [27, 28].

The article "Design of Public Building Space in Smart City Based on Big Data" was published in 2022. Journal: J Environ Public Health.

### 4.2. GIS Remote Sensing Feature Extraction of Spatial Information Changes of Public Buildings in Smart Cities

GIS can be divided into the following five parts: personnel is the most important part of GIS. Developers must define various tasks to be executed in GIS and develop processing programs. Skilled operators can usually overcome the shortcomings of GIS software functions, but the opposite is not true. The best software cannot make up for the negative effect brought by the operators' ignorance of GIS.

Data: accurate and available data can affect the results of query and analysis.

Hardware: the performance of hardware affects the processing speed of software to data, whether it is convenient to use and possible output mode.

The software includes not only GIS software but also various databases, drawing, statistics, image processing, and other programs.

Process: GIS requires clear definition and consistent methods to generate correct and verifiable results.

GIS is a kind of information system. The difference is that it can operate and process geo-referenced data. Geographic reference data describes the location and attributes of spatial elements on the Earth's surface (including the atmosphere and the shallow subsurface space). There are two geographical data components in GIS: spatial data, which is related to the geometric characteristics of spatial elements. Attribute data provides information about spatial elements.

According to the analysis results of spatial composition parameters of public buildings in smart cities, the spatial combination big data GIS information base of architectural structure aesthetics is analyzed in the polysemy morphological elements distribution of composite spaces. The output model of regularization parameters of GIS model base of spatial information changes of public buildings in smart cities is as follows:

(6) IGIS=ICN;DN|sN=∑i=1NhDi|si−hDi|Ci,si=∑i=1NhgiCi+Vi−hVi,

where *C*^*N*^ is the acquired massive spatiotemporal data of public buildings in smart cities, *D*^*N*^ is the spatial information data of public buildings in smart cities, *s*^*N*^ is the big data distribution of physical space, *N* is the data stock, *g*_*i*_ is the structural parameter of GIS remote sensing information, and *C*_*i*_ is the shape parameter of three-dimensional objects in public buildings in smart cities. *V*_*i*_ indicates the discrimination between the geometric spatial composition of public buildings in smart cities and some non-smart cities, and *h*(*V*_*i*_) indicates the probability density function for the regional parameters of the geometric spatial composition of public buildings in smart cities and some non-smart cities [29, 30].

The article "Design of Public Building Space in Smart City Based on Big Data" was published in 2022. Journal: J Environ Public Health.

Therefore, according to the analysis results of the spatial configuration parameters of public buildings in smart cities, the spatial combination big data GIS information base of architectural structure aesthetics is constructed, and the geometric features of public buildings in smart cities in towns and nature are considered, so that the change characteristics of spatial information of geometric features of public buildings in smart cities can be recognized.

## 5. Simulation and Test

The vertical spatial organization in public space composite design is to lead the urban space to the high-rise building, meet the space requirements of different functions under intensive layout, and form a good interaction between internal and external spaces. In essence, it is the expression of urban space changing from two-dimensional to three-dimensional layout. Vertical spatial organization has the following ways: multi-directional stacking, staggered stacking, vertical penetration, spatial embedding, and vertical stacking. Therefore, this paper proposes a smart city public building space design based on big data. Based on the above theoretical research, the following tests are designed to verify the proposed method.

### 5.1. Experimental Preparation

The experiment takes a city public building as the research object. Based on the Landsat 8 remote sensing image and sentinel 2 remote sensing image of the building, 100 sample points are selected on each ground feature.

The article "Design of Public Building Space in Smart City Based on Big Data" was published in 2022. Journal: J Environ Public Health.

On the basis of Table 1, the geometric spatial planning and color aesthetic positioning of smart city public buildings are carried out by the method of joint feature analysis of urban development and spatial layout, and the characteristic quantity of urban building integration morphological elements is extracted by the method of spatial composite aesthetic feature analysis of urban building structures. By calculating the fuzzy infiltration of spatial interface and the interactive change parameters of internal and external spaces, the spectral distribution ratio of geometric spatial information of smart city public buildings is obtained as shown in Table 2.

### 5.2. Test Results and Analysis

On the basis of the above parameter design and calculation, according to the calculation method of spatial composition index of public buildings in smart cities designed in this paper, the detected spatial GIS remote sensing image of public buildings in smart cities is obtained by using the method of GIS remote sensing detection, as shown in Figure 5.

There is interference in the remote sensing image in Figure 5. The method in this paper is used to extract the variation characteristics of the spatial information of the geometric form of public buildings in smart cities, and the extracted spatial composition and distribution characteristics of the geometric form of public buildings in smart cities are shown in Figure 6.

According to the analysis of Figure 6, this method can effectively suppress the cloud interference, set the cloud pixels as the background values, and accurately realize the feature recognition of the spatial information changes of public buildings in smart cities. The detection of spatial composition index of public buildings in smart cities is more robust. Finally, the spatial composition and color planning results of public buildings in smart cities are shown in Figure 7.

By analyzing Figure 7, it is known that the method in this paper has a good performance in detecting the changes of spatial information and identifying features of public buildings in smart cities, and has a good environmental adaptability.

Comprehensive analysis shows that the method in this paper has strong anti-interference ability, and can accurately identify the geometric shape and spatial change characteristics of public buildings in smart cities. At the same time, this method has good environmental adaptability, and can accurately detect the geometric spatial information and features. Therefore, after the method in this paper is applied to the space design of smart city public buildings, it can realize high-precision spatial combination big data extraction at the aesthetic level of building structure in a large area, and improve the spatial composition and color planning ability.

The article "Design of Public Building Space in Smart City Based on Big Data" was published in 2022. Journal: J Environ Public Health.

## 6. Conclusions

With the rapid development of urban compactness, urban public space is constantly being squeezed out, and the street interface has evolved from the original small-scale street-facing buildings with affinity to closed, cold, and large-scale residential areas and public buildings. The planned urban public spaces, such as parks and squares, are few in number, extensive in design and single in function, which makes it difficult to meet the diversified needs of urban residents' communication and leisure, commercial and cultural activities, etc. In this case, the public spaces inside and around the buildings gradually assume the role of urban public spaces, providing people with communication and activity venues. From the perspective of architectural space, the more complex and contradictory the needs to be met by the building, the more diverse and complex its spatial forms and combinations will be. Therefore, it has become an urgent problem to be solved how to break the singleness of the interior of the building through the composite design of the public space of the building, make it present more diverse spatial patterns and introduce behaviors suitable for contemporary society, and open up the public space inside and outside the building, so that it can be more introduced into urban functions.

This paper combines big data analysis technology and remote sensing image recognition technology to analyze the remote sensing parameters under the spatial feature distribution of public buildings in smart cities. Combined with the method of image feature analysis, the geometric form space composition and color planning and design of smart city public buildings are carried out. Based on the GIS remote sensing image analysis of the spatial combination change at the aesthetic level of the building structure, the big data extraction of the spatial combination at the aesthetic level of the building structure is realized. The experimental analysis shows that this method has high environmental adaptability and robustness to the spatial combination big data extraction of architectural structure aesthetics, and can realize high-precision spatial combination big data extraction of architectural structure aesthetics in a large area.

## Figures and Tables

**Figure 1:** Big data processing smart city public building space.

**Figure 2:** The geometric form and spatial composition of public buildings in smart cities and the technical route of color planning and design.

**Figure 3:** Construction of spatial composition index model of public buildings in smart cities.

The article "Design of Public Building Space in Smart City Based on Big Data" was published in 2022. Journal: J Environ Public Health.

**Figure 4:** Analysis process of gray value of spatial combination in architectural structure aesthetics.

**Figure 5:** Remote sensing image map.

**Figure 6:** Extraction results of geometric form and spatial composition characteristics of public buildings in smart cities. (a) Primitive character. (b) Vector range. (c) Edge feature extraction.

**Figure 7:** Geometry spatial composition and color planning of public buildings in smart cities.

**Table 1:** Remote sensing GIS data source information table (wavelength unit: nm).

Wave band	Landsat 8	Sentinel 2	GF-1
Blue band	0.149	0.236	0.7429
Green band	0.745	0.159	0.9226
Red band	0.393	0.593	0.7462
Near-infrared band	0.698	0.867	0.1791
Short wave	0.158	0.217	0.0484
Near-infrared 1 band	0.322	0.409	0.8456
Short-wave infrared band 2	0.733	0.090	0.7757

**Table 2:** Spectral distribution ratio of spatial information of public buildings in smart cities.

Ground feature structure of urban public building space	Q1	Q2	Q3	Q4	Q5	Q6
Spatial composition of geometric form of urban public buildings	0.306	0.284	0.693	0.723	0.306	0.284
Color composition of urban public buildings	2.638	0.792	0.301	0.409	2.638	0.792
Shadow	4.245	0.364	0.252	0.506	4.245	0.364
Afforestation	0.427	0.461	0.351	0.382	0.427	0.461
Energy conservation	5.761	0.912	0.138	0.985	5.761	0.912
Ground traffic	2.684	0.725	0.217	0.970	2.684	0.725
Network of underground	1.701	0.100	0.796	0.595	1.701	0.100
City block	4.271	0.209	0.728	0.158	4.271	0.209

## Data Availability

The raw data supporting the conclusions of this article will be made available by the authors, without undue reservation.
